# Comparison of a Minimally Invasive Tissue-Sparing Posterior Superior (TSPS) Approach and the Standard Posterior Approach for Hip Replacement

**DOI:** 10.1155/2022/3248526

**Published:** 2022-06-30

**Authors:** Matteo Romagnoli, Federico Raggi, Tommaso Roberti di Sarsina, Alvise Saracco, Marco Casali, Alberto Grassi, Stefano Zaffagnini

**Affiliations:** ^1^Ortopedia e Traumatologia Rizzoli-Argenta, IRCCS Istituto Ortopedico Rizzoli, Bologna, Italy; ^2^IIa Clinica Ortopedica e Traumatologica, IRCCS Istituto Ortopedico Rizzoli, Bologna, Italy; ^3^Dipartimento Rizzoli Sicilia, IRCCS Istituto Ortopedico Rizzoli, Bologna, Italy

## Abstract

**Purpose:**

The purpose of this study is to compare the functional and clinical outcomes, blood loss, complication rate, and hospital length of stay (LOS) of total hip replacement (THR) using a minimally invasive tissue-sparing posterior superior (TSPS) approach and the standard posterior approach.

**Materials and Methods:**

This retrospective, observational, double-centered study included 38 patients undergoing hip replacement. The patents were divided into two groups: control group (19 patients), who underwent surgery with the standard posterior approach, and treatment group (19 patients), who received the same type of implant with ceramic-on-ceramic bearing via the TSPS approach. Hemoglobin level was assessed preoperatively, on first and second postoperative days, and on discharge day. Harris hip score and Western Ontario and McMaster Universities Arthritis Index were used to measure the clinical and functional outcomes. Hospital LOS and incidence of early and late complications were assessed in both groups. Postoperative anteroposterior pelvis X-ray was performed to assess the correct positioning of implants.

**Results:**

Better early clinical outcomes (*p* = 0.0155), lesser blood loss (*p* < 0.0001), and reduced hospital LOS (*p* < 0.0001) were observed in the TSPS group than in the control group. No major adverse effects occurred in both groups, and a satisfactory implant orientation was achieved in all patients.

**Conclusions:**

The TSPS approach is a reliable minimally invasive procedure for THR as it allows an accurate orientation of the components and provides better early postoperative functional outcomes, faster recovery, significantly lower blood loss, and shorter hospital LOS than the standard posterior approach. However, further research is needed to confirm the promising results and cost-effectiveness of the TSPS approach in larger cohorts with a longer follow-up period.

## 1. Introduction

Correct implant positioning and effective soft tissue management are critical in total hip replacement (THR) to prevent complications and optimize outcome [1–3]. In recent years, minimally invasive surgery (MIS) techniques have gained increasing popularity due to minimal soft tissue and muscle damage around and of the hip through both smaller skin incision and fewer muscles splitting or detachment procedures, which are typically required in conventional approaches [3, 4]. In addition, less pain, less blood loss, faster recovery, and consequently shorter hospital length of stay (LOS) are associated with MIS in THR, although MIS may increase the duration of surgical procedure and the risk of perioperative complications [5, 6] due to a steeper learning curve as compared to standard procedures [7].

Capuano et al. [8] developed the tissue-sparing posterior superior (TSPS) approach, an MIS technique based on the standard posterior approach described by Moore [9], using the same proximal incision of 6–8 cm but avoiding the detachment of external rotator muscles, except the piriformis tendon, which is repaired at the end of the procedure, and the posterior capsule. The aim was to reduce blood loss from iatrogenic lesion of the medial circumflex artery, which typically occurs during sectioning of the external rotators in the standard posterior approach and to prevent complications such as dislocation [10–13] to gain a faster return to daily routine. Capuano et al. [8] reported better early postoperative outcomes and a faster postoperative recovery using the TSPS approach compared to the standard posterolateral approach [8]. However, they highlighted the need for further studies to confirm their preliminary findings. Therefore, in this study, we compared THR with ceramic-on-ceramic bearing via the minimally invasive TSPS approach and the standard posterolateral approach. The hypothesis was that the TSPS approach results in lesser blood loss, shorter LOS, and better outcome compared to the standard posterior approach.

## 2. Materials and Methods

Thirty-eight patients undergoing THR were included in the study. The patients were divided into two groups: control group (standard posterior approach, 19 patients) and treatment group (TSPS approach, 19 patients). TSPS approach was performed by a senior surgeon (M.R.) between June 2016 and February 2018 at the IRCCS Rizzoli Orthopaedic Institute after obtaining a signed informed consent. The inclusion criteria were primary hip osteoarthritis, avascular necrosis, and congenital dysplasia of the hip Crowe type I–II [14]. The exclusion criteria were patients with previous hip surgery or joint replacement, patients who lacked capacity to consent, <18 years of age, or those affected by any condition that may interfere with the THR survival or outcome, such as neurological disorders and body mass index (BMI) >35 kg/m^2^. In the control group, THR via the conventional posterior technique was also performed by the same surgeon within the same period. These patients fulfilled the same inclusion\exclusion criteria. The indication to perform TSPS technique rather than the conventional approach was not based on patients' characteristics or radiographic features.

### 2.1. Operative Technique

For the TSPS approach, the patient was placed in a lateral position on a standard surgical table. A correct vertical position of the pelvis was obtained by placing two cushions anterior and posterior to the pelvis. The greater trochanter was palpated, and skin incision was performed starting at two-thirds of the width of the greater trochanter from its anterior margin and extends for 6–8 cm, parallel to the fibers of the gluteus maximus. The length of the skin incision must be at least 1.5 times larger than the diameter of the femoral head, which was previously assessed by accurate preoperative planning (Figure 1). Subcutaneous fat and then the fascia lata were incised. The gluteus maximus was then split in line with its fibers with care to avoid cutting them. The gluteus medius muscle was located and divaricated. Then, the piriformis tendon was located and tagged with one hard suture and then detached using an electrocautery (Figure 2).

Longitudinal capsulotomy with a flap of the superior capsule was performed, exposing only the femoral head and carefully avoiding dislocation, which can lead to possible external rotator muscles rupture. The lesser trochanter was used as a reference point to perform an intraarticular neck resection of the correct length, according to the preoperative plan (Figure 3(a)). Schanz screw was used to excise the femoral head and was inserted in the most cranial direction possible while maintaining a cranial-caudal direction toward the neck. Then, with the leg in abduction to relax the gluteus muscles, the Schanz screw was turned in the cranial-caudal direction to extract the femoral head (Figure 3(b)).

Partial capsulectomy was performed, and the labrum was then excised to prevent any soft tissue impingement between the acetabulum and the implant. A dual-offset reamer handle was used for acetabular preparation. The final implant was then positioned employing a dual-offset impactor with 45° of abduction and 20°–25° of anteversion, using the transverse ligament as a landmark for the cup orientation. Osteophytes around the acetabulum were then removed. The femur was reamed with the upper leg oriented in maximum adduction but less internal rotation than the standard posterior approach. The definitive femoral stem was then positioned using a straight-handled impactor. Finally, the superior articular capsule was reconstructed, and tenorrhaphy of the piriformis tendon was performed [7, 8]. Patients in the control group underwent the standard posterior approach [9] without reconstruction of the capsule, whereas patients in the treatment group underwent surgery with the TSPS approach [8]. The fascia, subcutaneous layer, and skin were closed according to the surgeon's preferences using drainage in both groups. M.R performed all the procedures in both groups. An uncemented acetabular press-fit cup (Ti-Por; Adler Ortho S.R.L., Cormano, Italy) and a cementless short stem with metaphyseal grip (Pulchra; Adler Ortho S.R.L.) with a ceramic-on-ceramic bearing were implanted in all patients.

### 2.2. Postoperative Rehabilitation

Prior to the surgery, the patients were given a booklet regarding bed exercises. They were informed that isometric rehabilitation would be initiated immediately postoperation. Information regarding dislocation maneuvers that should be avoided and correct postures to maintain in bed were given. Partial weight bearing (up to 50% of the body weight), as tolerated by the patient, was permitted from postoperative day 1. Muscle strengthening exercises and functional reeducation of the hip were progressively introduced. Complete weight bearing was encouraged starting from postoperative day 15.

### 2.3. Patient Evaluation

Hemoglobin (Hb) level was assessed preoperatively, on postoperative day 1 and day 2, and on day of discharge. Blood loss was evaluated by calculating the difference between preoperative (expressed in g/dl) and postoperative Hb values at preoperative day 1. Blood transfusions recording the blood volume transfused were reported; the transfusion criteria were postoperative Hb level<8 g/dl or patient presenting symptoms of hypoperfusion even with Hb values between 8 and 9 g/dl [8]. Blood transfusions were decided by a doctor not involved in the study or the surgery and who was blinded to the surgical technique used. In both groups, we also evaluated the hospital LOS and incidence of early and late complications. The Harris hip score (HHS) [15] and Western Ontario and McMaster University Index (WOMAC) [16] were used to measure the clinical and functional outcome of patients preoperatively and at 4-month follow-up.

### 2.4. Radiographic Evaluation

All patients underwent a postoperative anteroposterior pelvis X-ray centered on the pubic symphysis, and the film-focus distance was 120 cm to assess the correct positioning of implants. The method by Lewinnek et al. [17] was used to calculate anteversion and to measure cup inclination. Anteversion was defined as arcsin (short axis/long axis) and inclination as the angle between the line on which the long axis of the ellipse is located and the inter-teardrop line.

With the picture archiving and communication system (PACS) program, the ellipse of the acetabular cup's opening rim was drawn; the short axis and long axis were determined and measured. Anteversion was calculated using the equation. Inclination was directly measured on a plain radiograph with the PACS program. The stem position was evaluated in the anteroposterior X-ray; varus alignment was defined as femoral stem alignment ≥5° on radiographic assessment with respect to the long axis of the femur.

Anteroposterior and lateral radiographs were repeated at 4 months to evaluate the stability of the implant according to Engh et al. [18] criteria for the stem and Udomkiat et al. [19] criteria for the acetabular cup.

### 2.5. Statistical Analysis

Statistical analysis was performed using MedCalc for Windows version 15.0 (MedCalc Software, Ostend, Belgium). Sample size was calculated using LOS as the primary outcome; using a power of 80% and alpha value of 0.05, 16 patients per group were needed to detect difference of 1 (±1) day. To overcome possible lost to follow-up of 15%, a total of 19 patients per group were included.

Continuous data were summarized using mean and standard deviation, while categorical data were expressed by percentages. The *t*-test for paired samples and the Fisher exact test were used to compare continuous data and categorical data, respectively, among the two groups. Multiple regression analyses were performed using the Hb levels on postoperative day 1 and day 2, blood loss (estimated as decreasing Hb count), hospital LOS, and outcome scores (HHS and WOMAC) at 4-month follow-up as dependent variables, whereas age, sex, American Society of Anesthesiologists score, BMI, surgical approach, preoperative clinical scores (HHS and WOMAC), and preoperative Hb level were considered as independent variables. The significance level was set at *α* = 0.05.

### 2.6. Ethics

In accordance with the Italian law, ethics committee approval was not obtained since the study was completely observational, with no changes to standard clinical practice [8]. The clinical study was conducted according to the Declaration of Helsinki.

## 3. Results

### 3.1. Patient Characteristics

A total of 38 patients (19 in the TSPS group and 19 in the control group) were included in the study. The two groups were homogeneous for clinical and demographic characteristics (Table 1). Mean preoperative Hb levels (g/dl) were comparable for both groups (*p* = 0.1295), including the average preoperative HHS (*p* = 0.8129) and average preoperative WOMAC (*p* = 0.5192) (Table 1).

### 3.2. Clinical Results

In both groups, no patients were lost to follow-up, and no serious adverse events directly related to the procedures occurred. However, hospital LOS was significantly shorter in the TSPS group (*p* < 0.0001), higher Hb levels on postoperative day 1 (*p* = 0.0178), and lesser blood loss, estimated as decreasing Hb count between preoperative and postoperative day 1, (*p* < 0.0001) as compared to the control group (Table 2).

However, differences between Hb levels on postoperative day 2 (*p* = 0.0942) and blood transfusions (*p* = 1.0000) were not statistically significant. According to the multiple regression analysis, patient age (*p* = 0.03), preoperative Hb levels (*p* < 0.0001), and surgical approach (*p* < 0.0001) were significant predictors of Hb levels on both postoperative day 1 and day 2, as well as for blood loss (Table 3). In addition, the TSPS approach was the only significant predictor of shorter LOS (*p* < 0.0001). The HHS and WOMAC score significantly improved from the preoperative status to the 4-month follow-up in both groups (*p* < 0.05). No significant differences were found between both groups regarding the 4-month follow-up values of both HHS (*p* = 0.1024) and WOMAC (*p* = 0.0685) score (Table 2). However, according to the multiple regression analysis, the TSPS approach was the only significant predictor of higher values of WOMAC score (*p* = 0.0155) (Table 4). No predictors were found for postoperative HHS.

### 3.3. Radiographic Results

The radiographic evaluation of implant positioning postoperatively was carried out by the same surgeon (M.C.) for all cases. The average cup inclination was 41.9° ± 2.2° (range 36.1°–44.8°) in the TSPS group and 40.6° ± 2.2° (range 36.5°–44.6°) in the standard posterolateral approach group, with no significant differences (*p* = 0.6768). No significant differences (*p* = 0.3619) were reported for cup anteversion, with an average value of 21.2° ± 1.9° (range 17.7°–24.2°) in the TSPS group and 20.7 ± 1.4 (range 18.1°–21.1°) in the standard posterolateral group. All the cups in both groups were within the “safe zone” of 15° ± 10° for anteversion and 40° ± 10° for inclination.

The evaluation of the stem alignment showed no significant differences (*p* = 0.8966), with an alignment of 2.4° ± 2.5° (range -3.4° to 8.5°) in the TSPS group and 2.5° ± 2.2° (range -2.1° to 5.9°) in the standard posterolateral group. Moreover, only two patients in each group had stem positioned with a varus alignment >5°. Anteroposterior X-ray and lateral X-ray at 4-month follow-up showed no signs of loosening of the stem or acetabular cup in both groups (Figures 4(a)–4(d)).

## 4. Discussion

The most important finding of the present study was that the TSPS approach was associated with lesser blood loss both intraoperatively and postoperatively as compared to the standard posterolateral approach. Consequently, this leads to shorter hospital LOS. Based on the regression analysis, the TSPS surgical approach was the only predictor of shorter LOS. Lesser blood loss may reduce pain, cardiac complications, and hematoma formation, consequently resulting in slower rehabilitation, wound breakdown, infection, and blood transfusions [8, 20–22].

In our study, only one patient treated with the TSPS approach required blood transfusion as compared to four patients treated with the conventional technique. However, due to the small sample size of our study, this finding was not significant. In addition, the reduced blood loss may have likely affected the hospital LOS, which was significantly shorter in the treatment than in the control group. Short hospital stays are associated with decreased health-care costs for health-care services, as reported by a previous study that approximately US$4,000 per patient is saved when using MIS instead of conventional surgeries [23].

A higher short-term WOMAC score and HHS were reported in the TSPS group, indicating a better early clinical outcome that may affect the rehabilitation program, which may lead to a shorter recovery. Regarding functional outcomes, based on the regression analysis, the TSPS surgical approach was the only predictor of a high WOMAC score. Nevertheless, according to a previous study, the WOMAC score tends to be comparable to the other standard approaches in a mid-term evaluation [24].

Compared to Capuano et al. [8], despite the smaller sample size in the present study, the bias related to the variety of implant designs and bearing of their study has been overcome. In the present study, the same uncemented acetabular press-fit cup (Ti-Por; Adler Ortho S.R.L., Cormano, Italy) and a cementless short stem with metaphyseal grip (Pulchra; Adler Ortho S.R.L., Cormano, Italy) with ceramic-on-ceramic bearing have been used for both groups. Furthermore, we gained a satisfactory implant orientation in both groups, meaning that a less invasive TSPS approach does not affect the positioning of the components when compared to the larger exposure of the conventional posterior approach. No adverse event occurred in either group; however, in the authors' opinion, the shorter LOS and higher short-term functional scores could be related to the less invasiveness of the TSPS approach, reinserting the piriformis muscle and preserving the articular capsule that could lead to a longer follow-up to fewer cases of hip dislocation; however, further research is needed to verify this.

We believe that the positive findings of our study are even more significant as all the TSPS procedures performed in this study have been performed by the main author at the beginning of his learning curve, which includes almost 50 cases or 25–30 cases if the surgeon is familiar with the standard posterior approach [8]. Compared to other popular MIS approaches, such as the MIS anterior approach described by Lesur and Laude [25], the TSPS technique has the main advantage of not requiring a special surgical table. This approach can be easily converted to a conventional posterior approach at any time during the surgery, with the possibility of both a proximal extension toward the iliac crest to the ilium and a distal extension to the femoral shaft by splitting or elevating the vastus lateralis from the lateral intermuscular septum.

This study has several limitations. First is the small sample size. However, a preliminary study was needed to set the foundation for further research. Moreover, since a power analysis was performed using LOS as the primary outcome, the study could result underpowered to assess other outcomes such as the number of transfusions, WOMAC score, or HHS. Second is the nonrandomized design due to the need for a pilot study involving the first patients who underwent a new surgical technique that was never described previously. Thus, in our opinion, it is not ethically and methodologically accurate to be proposed within a randomized clinical trial. Nevertheless, sample design and cohort selection were assessed using the same inclusion criteria for both groups to reduce the risk of selection bias. Moreover, the small sample size was insufficient to identify other possible advantages, or it limits the external validity. However, the sample size was determined based on the nature of this research as a “pilot” study to assess the effectiveness of the TSPS approach by an unbiased surgeon, which is independent of the developer of the technique. Due to the promising initial results, the technique has been introduced in the surgical routine, and further studies with larger sample cohorts and longer follow-ups are needed to confirm these findings.

Another limitation is that no gate analysis nor muscular strength assessment was performed, as it was not part of our standard postoperative protocol following a THA. Finally, the short-term follow-up of 4 months does not allow us to draw a definitive conclusion regarding neither the mid- to long-term outcomes of this procedure nor the implant survivorship, which should be investigated in further studies with longer follow-ups. Meanwhile, the findings of the present study support the safety of the TSPS approach, the ability to properly position the implants despite the soft tissue mini-invasivity, and a limited benefit for early recovery.

## 5. Conclusions

The TSPS approach has a demonstrable advantage over the standard posterior approach for THR as it allows an accurate orientation of the components and provides better early postoperative functional outcomes, faster recovery, significantly lower blood loss, and, consequently, reduced hospital LOS than the standard posterior approach. However, further research is needed to confirm the promising results and cost-effectiveness of the TSPS approach in larger cohorts with a longer follow-up period.

## Figures and Tables

**Figure 1:** The patient is placed in a lateral position on a standard surgical table. The greater trochanter is palpated, and skin incision is performed starting at two-thirds of the width of the greater trochanter from its anterior margin and extends for 6–8 cm. The length of the skin incision must be at least 1.5 times larger than the diameter of the femoral head.

**Figure 2:** The piriformis tendon is located and tagged with one hard suture and then detached using an electrocautery.

**Figure 3:** The lesser trochanter is used as a reference point to perform an intraarticular neck resection of the correct length, according to the preoperative plan (a). Schanz screw is used to excise the femoral head and is inserted in the most cranial direction possible while maintaining a cranial-caudal direction toward the neck. With the leg in abduction to relax the gluteus muscles, the Schanz screw is turned in the cranial-caudal direction to extract the femoral head (b).

**Figure 4:** Radiographic images of the TSPS (a, b) and posterior (c, d) group. (a, c) Preoperative AP radiographs of the pelvis with the calibration for the planning. (b, d) Postoperative radiograph which shows the correct implant placement.

**Table 1:** Demographic characteristics of the patients.

Characteristics	Posterior approach (*n* = 19)	TSPS approach (*n* = 19)	*p* value
Sex (M/F)	11/8	15/4	0.2952
Age at surgery (y)	56.2 ± 10.7	57.3 ± 11.5	0.7724
Side (R/L)	11/8	10/9	1.0000
BMI (kg/m^2^)	26.2 ± 3.2	26.7 ± 2.9	0.5990
ASA classification (grade)			0.4612
I	6 (32%)	4 (21%)	
II	13 (68%)	14 (74%)	
III	0 (0%)	1 (5%)	
Preoperative HHS	36.8 ± 11.0	37.8 ± 14.2	0.8129
Preoperative WOMAC	74.4 ± 17.6	69.9 ± 24.2	0.5192

Statistically significant comparisons (*p* < 0.05) are marked in bold and with ∗. Abbreviations: TSPS: tissue-sparing posterior superior; M: males; F: females; R: right; L: left; BMI, body mass index; ASA: American Society of Anesthesiologists; HHS: Harris hip score; WOMAC: Western Ontario and McMaster Universities Arthritis Index.

**Table 2:** Postoperative and follow-up evaluation.

	Posterior approach (*n* = 19)	TSPS approach (*n* = 19)	*p* value
LOS (days)	7.0 ± 2.2	3.8 ± 1.3	0.0001∗
Hb postoperative day 1 (g/dl)	10.7 ± 1.2	11.7 ± 1.3	0.0178∗
Hb postoperative day 2 (g/dl)	9.9 ± 1.6	10.8 ± 0.9	0.0942
Blood loss (g/dl)	3.8 ± 1.1	2.1 ± 0.8	0.0001∗
Transfusion (Y/N)	4/15	1/18	0.1499
4-month HHS	86.2 ± 8.2	90.6 ± 8.3	0.1024
4-month WOMAC	13.1 ± 10.7	7.4 ± 7.7	0.0685

Statistically significant comparisons (*p* < 0.05) are marked in bold and with ∗. Abbreviations: TSPS: tissue-sparing posterior superior; LOS: length of stay; R: right; L: left; Hb: hemoglobin; HHS: Harris hip score; WOMAC: Western Ontario and McMaster Universities Arthritis Index.

**Table 3:** Multiple regression analysis considering postoperative day 1 and day 2 Hb levels and LOS as the main outcomes.

Variables	Hb						LOS (days)		
	Day 1 (g/dl)			Day 2 (g/dl)					
	Coeff	SE	*p* value	Coeff	SE	*p* value	Coeff	SE	*p* value
Age (y)	+0.034	0.015	0.0300∗	+0.003	0.022	0.9051	-0.014	0.035	0.6821
Sex (F)	-0.318	0.354	0.3762	-0.473	0.655	0.4807	-0.554	0.824	0.5068
ASA classification	-0.304	0.361	0.4057	+0.386	0.577	0.5130	+0.488	0.840	0.5659
BMI (kg/m^2^)	-0.072	0.050	0.1588	-0.072	0.071	0.3234	+0.071	0.117	0.5455
TSPS approach	-1.410	0.296	0.0001∗	-1.539	0.467	0.0046∗	+3.580	0.690	0.0001∗
Preoperative Hb (g/dl)	+0.659	0.120	0.0001∗	+0.783	0.206	0.0015∗	-0.382	0.288	0.1831

Statistically significant predictors (*p* < 0.05) are marked in bold and with ∗. Abbreviations: Coeff: coefficient; SE: standard error; F: female; Hb: hemoglobin; LOS: length of stay; F: female; BMI: body mass index; TSPS: tissue-sparing posterior superior; ASA: American Society of Anesthesiologists.

**Table 4:** Multiple regression analysis considering HHS and WOMAC score at 4-month follow-up as the main outcomes.

Variables	4-month HHS			4-month WOMAC		
	Coeff	SE	*p* value	Coeff	SE	*p* value
Age (y)	+0.103	0.156	0.5125	-0.206	0.162	0.2144
Sex (F)	+2.641	3.700	0.4809	-6.874	3.817	0.0817
ASA classification	+1.044	3.782	0.7843	+3.467	3.976	0.3902
BMI (kg/m^2^)	-0.238	0.490	0.6301	-0.523	0.542	0.3424
TSPS approach	-5.733	3.106	0.0748	+8.417	3.279	0.0155∗
Preoperative Hb	+1.053	1.262	0.4105	-1.456	1.322	0.2795
Preoperative HHS	-0.111	0.123	0.3727	NA	NA	NA
Preoperative WOMAC	NA	NA	NA	-0.103	0.078	0.1943

Statistically significant predictors (*p* < 0.05) are marked in bold and with ∗. Abbreviations: Coeff: coefficient; SE: standard error; F: female; ASA, American Society of Anesthesiologists; BMI: body mass index; TSPS: tissue-sparing posterior-superior; Hb: hemoglobin; HHS: Harris hip score; WOMAC: Western Ontario and McMaster Universities Arthritis Index.

## Data Availability

The data of this study are available upon request.
